# Identification of Visual Imagery by Electroencephalography Based on Empirical Mode Decomposition and an Autoregressive Model

**DOI:** 10.1155/2022/1038901

**Published:** 2022-01-30

**Authors:** Yunfa Fu, Zhaoyang Li, Anmin Gong, Qian Qian, Lei Su, Lei Zhao

**Affiliations:** ^1^Faculty of Information Engineering and Automation, Kunming University of Science and Technology, Kunming 650500, China; ^2^Brain Cognition and Brain–Computer Intelligence Integration Group, Kunming University of Science and Technology, Kunming 650500, China; ^3^School of Information Engineering, Chinese People's Armed Police Force Engineering University, Xi'an 710000, China; ^4^Faculty of Science, Kunming University of Science and Technology, Kunming 650500, China

## Abstract

The traditional imagery task for brain–computer interfaces (BCIs) consists of motor imagery (MI) in which subjects are instructed to imagine moving certain parts of their body. This kind of imagery task is difficult for subjects. In this study, we used a less studied yet more easily performed type of mental imagery—visual imagery (VI)—in which subjects are instructed to visualize a picture in their brain to implement a BCI. In this study, 18 subjects were recruited and instructed to observe one of two visual-cued pictures (one was static, while the other was moving) and then imagine the cued picture in each trial. Simultaneously, electroencephalography (EEG) signals were collected. Hilbert–Huang Transform (HHT), autoregressive (AR) models, and a combination of empirical mode decomposition (EMD) and AR were used to extract features, respectively. A support vector machine (SVM) was used to classify the two kinds of VI tasks. The average, highest, and lowest classification accuracies of HHT were 68.14 ± 3.06%, 78.33%, and 53.3%, respectively. The values of the AR model were 56.29 ± 2.73%, 71.67%, and 30%, respectively. The values obtained by the combination of the EMD and the AR model were 78.40 ± 2.07%, 87%, and 48.33%, respectively. The results indicate that multiple VI tasks were separable based on EEG and that the combination of EMD and an AR model used in VI feature extraction was better than an HHT or AR model alone. Our work may provide ideas for the construction of a new online VI-BCI.

## 1. Introduction

Brain–computer interfaces (BCIs) represent revolutionary human–computer interactions that aim to bypass peripheral nerves and muscles of the spinal cord and neuromusculature to realize direct communication and control between brains and the outside world. This technology is expected to provide an alternative new communication or control method for patients with severe movement disabilities or for healthy people with ad hoc needs for BCIs.

BCIs based on imagery represent an important type of BCI [1]. The traditional imagery task is motor imagery (MI) [2, 3], which requires subjects to imagine moving a certain part of their body from a first-person perspective [4, 5]. MI is difficult for subjects and requires a certain amount of training, and approximately 20% of individuals are incapable of MI [6]. Hence, MI may not be the best mental task for controlling BCIs [1]. Compared with the properties of MI, visual imagery (VI) is another mental-imagery task that is easier to complete, and it consists of instructing subjects to visualize a picture clearly in their brain from a third-person perspective [4]. Such mental-imagery activity usually does not require training or only requires a small amount of training. However, compared to the number of studies on MI-BCIs, much less research has been conducted on VI-BCIs. Therefore, there is a need for more research on VI-BCIs.

Currently, VI-BCI studies [1, 4, 7–9] exhibit continued issues with VI task design, as indicated by results revealing a lack of significant differences between different VI tasks, which may make it difficult to distinguish electroencephalography (EEG) characteristics induced by differentially designed VI tasks. Compared with the selection and execution of MI tasks, VI tasks are widely selected and consist of any picture or scene from daily life. For example, Kosmyna et al. [1] chose a flower and a hammer as VI tasks, with an average classification accuracy of 52%. This result may be because the VI tasks that were selected were all static, resulting in poor separability of evoked EEG signals. Azmy and Safri [7] analyzed the maximum power difference between EEGs during the resting state and a VI task (i.e., imagining a star rotating clockwise), which showed that there was no significant difference between the two states; unfortunately, the classification accuracy was not reported. Neuper et al. [4] measured EEGs during resting states and while subjects were instructed to imagine their hands in a VI task, which yielded an average classification accuracy of 56%. Koizumi et al. [8] used EEG to classify VI tasks of an unmanned aerial vehicle (UAV) moving in three planes (up/down, left/right, and front/back), with an average classification accuracy of 84.6% in prefrontal cortex. Sousa et al. [9] used EEG to classify three types of VI tasks: static points, dynamic points moving vertically in the up and down directions, and dynamic points moving vertically in the up, down, left, and right directions; this study yielded an average classification accuracy of 87.64%. Collectively, the above static VI task designs led to poor separability of evoked EEG signals, whereas use of a combination of moving VI tasks led to better separability of evoked EEG signals. Hence, the aim of this study was to combine static VI tasks (static pictures of visual imagery) and moving VI tasks (dynamic pictures of visual imagery), with the hypothesis that the EEG characteristics induced by these two different VI tasks would be separable.

In addition, the classification accuracies resulting from the feature-extraction methods used by previous VI-BCI studies could be improved [1, 4, 8, 9]. Kosmyna et al. [1] extracted power-spectrum features of EEG signals related to two VI tasks—flower and hammer—using a classifier based on spectrally weighted common spatial patterns, which yielded a low classification accuracy (52%). Neuper et al. [4] extracted frequency-band features of EEG signals related to two VI tasks, hand movement, and resting state, using a classifier based on distinction-sensitive learning vector quantization, which yielded a low-average classification accuracy (56%). Koizumi et al. [8] extracted power-spectral density features of the frequency bands of EEG signals related to three types of VI tasks and used a classifier based on a support vector machine (SVM), which yielded a moderate classification accuracy of 84.6%. Sousa et al. [9] extracted power-spectrum energy features of EEG signals related to three types of VI tasks and used an SVM classifier, which yielded a moderate classification accuracy of 87.64%. In contrast to these previous studies, our study used a combination of moving and static VI tasks to determine the resultant classification accuracies based on Hilbert–Huang Transform (HHT), autoregressive (AR) models, a combination method of empirical mode decomposition (EMD) and AR models for feature extraction, and an SVM for classification.

EMD has been used in HHT. HHT is an effective time–frequency analysis method for nonlinear and nonstationary signals [10]. Considering the nonlinear and nonstationary characteristics of EEG signals, some research has applied HHT to MI-BCIs, which has yielded promising results [11–14]. Some research also used the improved algorithm for empirical mode decomposition to classify motor imagery or other types of EEG signals such as epilepsy or depth of anesthesia [15–18]. However, this method has not yet been used in VI-BCIs. The AR model is a method for time-series analysis, and it has been used in MI-BCIs [19, 20]. AR model parameters gather important information, and studies have shown that the autoregressive parameters of AR model are most sensitive to state-dependent changes [21–23]. Therefore, autoregressive parameters of the AR model have been used as eigenvectors to represent EEG changes related to the state of subjects, which has yielded promising results [19, 20]. A combination of the EMD and the AR model is commonly used in mechanical fault diagnosis [24–26]. Zhang et al. investigate feature extraction of electroencephalogram (EEG) based emotional data by focusing on empirical mode decomposition (EMD) and autoregressive (AR) model to classify those emotional states. This combination has also yielded promising results [27]. It first uses EMD to decompose nonlinear nonstationary signals to obtain stable intrinsic mode function (IMF) components and then establishes the AR model for each IMF component. However, the combination of the EMD and the AR model has not been used for EEG feature extraction and classification verification of VI. Therefore, our study evaluated the HHT, the AR model, and a combination of the EMD and the AR model for their efficacies in classification accuracies of a novel VI-BCI paradigm.

## 2. Methods

### 2.1. Subjects, Visual Imagery Tasks, Time Sequences, Trials, and Experimental Settings

#### 2.1.1. Subjects

Eighteen right-handed subjects (male, 24–28 years old) participated in this study. All subjects had no perceptual or cognitive impairments, and their vision was either normal or corrected to normal via corrective lenses. Each subject signed an informed consent before the experiment.

#### 2.1.2. Visual Imagery Tasks

Previous VI-BCI studies that have used static pictures as mental tasks have resulted in poor separability of EEG characteristics [1]. In contrast, studies that have used MI as mental tasks have yielded separable characteristics of evoked EEGs. In this study, we used static-picture VI and moving-picture VI as mental task pairs. It is assumed that these two types of VI tasks can induce significantly different EEG characteristics. In our study, one VI task consisted of visually imagining a star with a static picture, while the other VI task involved visually imaging a star moving to the right, as shown in Figure 1.

#### 2.1.3. The Time Sequence and Process of Each Trial

The time sequence of a trial is shown in Figure 2. The subjects were required to first conduct a visual observation and then imagine a cued picture. When *t* = 0 s, the screen showed the following text: “the experiment is about to start.” This required the subjects to remain awake and relax for 3 s. When *t* = 3 s, a static star or a star moving to the right was randomly displayed on the screen. The subjects were required to observe and memorize the picture for 4 s. When *t* = 7 s, the cued picture disappeared and the screen went black. The subjects were required to visualize the picture just cued for 4 s. When *t* = 11 s, “rest” appeared on the screen for 5 s. After the rest period, the next trial was started. Each subject executed 200 trials, and each task consisted of 100 trials.

#### 2.1.4. Experimental Settings

The EEG equipment that was used is NT9200, and the sampling rate was 1,000 Hz. The electrode cap had 32 channels (according to the international 10–20 system), the grounding electrode was GND, the reference electrodes consisted of A1 and A2, and the electrode impedance was kept below 10 kΩ. A band-pass filter was set at 0.1 Hz and 100 Hz, and a 50 Hz notch filter was used to avoid power line noise. EEG data from eight channels—including FP2, F8, C3, CZ, C4, O1, Oz, and O2—were collected in this study.

### 2.2. Data Preprocessing

First, each EEG signal was linearly corrected to eliminate linear artifacts. Then, the original EEG signal was filtered with an elliptical filter with a digital band-pass filter at 8–13 Hz. The band-pass attenuation was 0.5 dB, and the stop-band attenuation was 50 dB. Finally, independent component analysis (ICA) was used to remove eye movement artifacts, ECG artifacts, and EMG artifacts.

### 2.3. Empirical Mode Decomposition and HHT

EMD is an adaptive signal time–frequency processing method that was creatively proposed by Huang et al. in 1998 [28]. Specifically, EMD is an adaptive data processing or excavation method that is suitable for the analysis of nonlinear and nonstationary time series. EMD assumes that any signal is composed of different IMFs, and each IMF can be linear or nonlinear. Each IMF component must satisfy two conditions [29]: (1) that the number of its extreme points and zero crossing points are the same or at most different by only one point and (2) that its upper and lower envelopes are locally symmetric with respect to the time axis. Any signal can be decomposed into a finite sum of IMFs, and the decomposition process should be based on the following assumptions [30]: (1) the signal has at least one maximum value and one minimum value; (2) the time-domain characteristics are determined by the extreme value interval; and (3) if the data sequence lacks the extreme value but contains the inflection point, the extreme point can be obtained by derivation.

The decomposition process of EMD is as follows [30]:

Step 1: all the maximum points of the original data series *x*(*t*) are determined, and a cubic-spline interpolation function is used to fit the upper envelope of the original data; then, all the minimum points are determined, and a cubic-spline interpolation function is used to fit all the minimum points to form the lower envelope of the data. The mean values of the upper and lower envelope are recorded as *m*_1_, and the average envelope *m*_1_ is then subtracted from the original data series *x*(*t*) to yield a new data series, *h*_1_:
  (1) $$\begin{array}{c} x\left(t\right)-m_{1}=h_{1}. \end{array}$$
In an ideal case, if it is an IMF, then it is the first component of *x*(*t*).
Step 2: if *h*_1_ does not satisfy the conditions of an IMF, *h*_1_ is used as the original data, Step 1 is repeated to obtain the average value of *m*_11_ of the upper and lower envelope lines, and then it is determined whether *h*_1(*k* − 1)_ − *m*_1*k*_=*h*_1*k*_ satisfies the conditions of IMF. If not, the cycle is repeated *k* times to get *h*_1(*k* − 1)_ − *m*_1*k*_=*h*_1*k*_, so that *h*_1*k*_ satisfies the conditions of IMF. Note that for *c*_1_=*h*_1*k*_, *c*_1_ is the first IMF component of signal *x*(*t*). Then, *c*_1_ is separated from *x*(*t*) to obtain the following:
  (2) $$\begin{array}{c} r_{1}=x\left(t\right)-c_{1}. \end{array}$$

Step 1 and Step 2 are then repeated with *r*_1_ as the original data to obtain the second IMF component *c*_2_ of *x*(*t*). This cycle is repeated *n* times to obtain *n* IMF components, as follows:

(3) $$\begin{array}{c} \left(\begin{array}{c} r_{1}-c_{2}=r_{2}\\ \vdots \\ r_{n-1}-c_{n}=r_{n} \end{array}\right). \end{array}$$

When *r*_*n*_ becomes a monotone function from which an IMF component can no longer be extracted, the cycle ends. From (2) and (3), we obtain the following:

(4) $$\begin{array}{c} x\left(t\right)=\overset{n}{\underset{j=1}{\sum }}c_{j}+r_{n}. \end{array}$$

Therefore, any signal *x*(*t*) can be decomposed into the sum of *n* IMF components and a residual *r*_*n*_, where the IMF component *c*_1_, *c*_2_,…, *c*_*n*_ contains the components of different frequency ranges from high to low, and they are all stable.

After EMD decomposition, Hilbert spectrum analysis was carried out, and Hilbert spectrum transformation was carried out for each IMF component according to the following formula:

(5) $$\begin{array}{c} y_{j}\left(t\right)=\frac{1}{\pi }\int_{-\infty }^{+\infty }\frac{c_{j}\left(\tau \right)}{t-\tau }\text{d}\tau . \end{array}$$

The analytical signal is as follows:

(6) $$\begin{array}{c} z_{j}\left(t\right)={\text{c}}_{\text{j}}\left(t\right)+iy_{j}\left(t\right)={\text{a}}_{\text{j}}\left(t\right)e^{i\theta_{j}\left(t\right)}. \end{array}$$

Furthermore, the instantaneous amplitude and phase can be obtained as follows:

(7) $$\begin{array}{c} a_{j}\left(t\right)=\sqrt{c_{j}{\left(t\right)}^{2}+y_{j}{\left(t\right)}^{2}},\\ \theta_{j}\left(t\right)=\text{arctan}\frac{y_{j}\left(t\right)}{c_{j}\left(t\right)}. \end{array}$$

In this study, an HHT transform was used to extract the average instantaneous energy as the eigenvector. First, EMD was used to decompose each EEG signal under each task. Then, the spectrum of each IMF component was analyzed by the Hilbert transform. The average instantaneous energy of the HHT amplitude was calculated, and the eigenvector was constructed. Finally, SVM was used to classify the test set.

### 2.4. AR Model

For general random signals, the AR model can be described as follows:

(8) $$\begin{array}{c} y\left(i\right)=\overset{p}{\underset{j=1}{\sum }}\phi_{j}y\left(i-j\right)+n\left(i\right), \end{array}$$

where *y*(*i*) is the *i*th sampling value of the signal, *ϕ*_*j*_ is the *j*th coefficient of the AR model, *n*(*i*) is the residual of white noise, and *p* is the order of the AR model.

In this study, the order of the AR model was first determined by the Akaike information criterion (AIC), and the optimal order of the AR model was with a *p* of 6. Then, the Burg algorithm was used to extract the six-order AR model coefficient (AR1,…, AR6), which was composed of 12-dimensional feature vectors: {*FP*2_*AR*1_,…, *FP*2_*AR*6_, *F*8_*AR*1_,…, *F*8_*AR*6_}. Finally, SVM was used to classify the test set.

### 2.5. Combination of EMD and AR Model

We first decomposed the VI-based EEG signals by EMD and obtained several stable IMF components. Then, we built the AR model for each IMF component and used the autoregressive parameters of the AR model and the variance of the residual as the eigenvector.

The EMD method was used to decompose the collected EEG signal *x*(*t*) to obtain *n* IMF components, *c*_1_(*t*), *c*_2_(*t*),…*c*_*n*_(*t*). Each IMF component contained different feature-scale information. Thus, through EMD analysis, the features of signal *x*(*t*) were completely described by these *n* IMF components, *c*_1_(*t*), *c*_2_(*t*),…*c*_*n*_(*t*). Therefore, through the feature extraction of *c*_1_(*t*), *c*_2_(*t*),…*c*_*n*_(*t*), the features of the original signal *x*(*t*) were obtained.

For any IMF component *c*_*i*_(*t*), the following autoregressive (AR) model (*m*) was established:

(9) $$\begin{array}{c} c_{i}\left(t\right)+\overset{m}{\underset{k=1}{\sum }}h_{ik}c_{i}\left(t-k\right)=e_{i}\left(t\right), \end{array}$$

where *h*_*ik*_ is the AR (*m*) model parameter of component *c*_*i*_(*t*); *m* is the model order; and *e*_*i*_(*t*) is the residual of the model, which is the white noise sequence with a mean value of 0 and variance of *e*_*i*_^2^. Therefore, *h*_*ik*_(*k*=1,2,…*m*) and *e*_*i*_^2^ can be used as feature vectors *A*_*i*_={*h*_*i*1_, *h*_*i*2_, ⋯*h*_*im*_, *e*_*i*_^2^} to identify VI tasks.

The steps of feature extraction with EMD combined with the AR model are as follows: Under the VI tasks of static and moving pictures, *n* samples were taken and 2*n* EEG signals were obtained as samples. EMD decomposition was carried out for EEG signals under each task. The number of IMF components obtained by different EEG signals was *n*_1_, *n*_2_,…*n*_2*N*_, and the maximum value in *n*_1_, *n*_2_,…*n*_2*N*_ was assumed to be *n*. If the number of IMF components in a sample was *n*_*k*_ < *n* (*k* = 1, 2, 2*n*), the zero vector was supplemented to have *n* components *c*_1_(*t*), *c*_2_(*t*),…*c*_*n*_(*t*), namely, *c*_*i*_(*t*)={0}(*i*=*n*_*k*_+1,  *n*_*k*_+2,…, *n*).

Each IMF component was energy-normalized to yield a new component $\bar{c_{i}\left(t\right)}$ as follows:

(10) $$\begin{array}{c} \bar{c_{i}\left(t\right)}=\frac{c_{i}\left(t\right)}{\sqrt{\int_{-\infty }^{\infty }c_{i}^{2}\left(t\right)\text{d}t}}. \end{array}$$

The AR model was established for each energy-normalized component $\bar{c_{i}\left(t\right)}$, and the order *m* of the model was determined by the final prediction error (FPE) criterion. The autoregressive parameter *h*_*ik*_(*k*=1,2,…*m*) and the residual variance *e*_*i*_^2^ of the model were estimated by the least-square method, and *h*_*ik*_ represented the *k*th autoregressive parameter of the *i*th IMF component.

The average value $\bar{h_{ik}}\left(k=1,2,\ldots ,m\right)$, $\bar{e_{i}^{2}}$ of *h*_*ik*_(*k*=1,2,…*m*), and *e*_*i*_^2^ of N samples in the same state were calculated, and $\bar{h_{ik}}$ and $\bar{e_{i}^{2}}$ were taken as the template eigenvector $\bar{A_{j,i}}=\left[\bar{h_{i1}},\bar{h_{i2}},\ldots ,\bar{h_{im}},\bar{e_{i}^{2}}\right]$ of the *i*th component, where *j* = 1, 2 represent the VI static picture and VI moving picture, respectively.

### 2.6. Support Vector Machine

SVM is a classification algorithm that improves the generalizing ability of learning machines by seeking the minimum structural risk and also minimizes the empirical risk and confidence range, so as to achieve sufficient statistical power for small samples [31].

The cores of the SVM algorithm that we used are as follows [32]: (1) in the case of linear separability, the learning strategy of interval maximization was used to find a hyperplane with the largest interval; (2) in the case of online separability, the feature vector of a low dimension was mapped to a high dimension by a kernel function to determine linear separability. The EEG signals we collected were small and nonlinear, so this SVM classifier was suitable for our present study.

The EEG data of FP2 and F8 were analyzed. The VI data consisted of 100 training datasets and 100 test datasets, including the labels of training samples and test samples. First, the training samples and labels were used to train the model. Then, the model was used to predict the labels of the test samples. Finally, the prediction labels were compared with the real labels to determine the classification accuracies.

## 3. Results

Table 1 shows the *t*-test value and variance analysis *p* value during the two VI tasks in each frequency band of the eight EEG channels. There were three variance analysis factors: (1) the VI tasks of imagining static and moving pictures; (2) the frequency-band range of the EEG signals (delta, theta, alpha, beta, and gamma); and (3) the EEG electrode channels (eight channels). The significance level was set as *p* < 0.05. The *t*-test results of the two VI tasks are shown in Table 1. The table also includes the *p* value and d*f* value of each electrode position obtained from the analysis of variance. As can be seen from the table, the most significant difference was in the *α* bands of FP2 and F8 (*p* < 0.001). In addition, a *t*-test was carried out to determine which channel had a significant difference. The results showed that the *p* values of positions F8 and FP2 were less than 0.01, which meant that there was a 99% significant difference between the data groups, which was the highest among all of the results.

The variance contribution rate and correlation coefficient of each IMF were calculated for IMF screening, as shown in Table 2. The sum-of-variance contribution rate of the first four stages of IMF was 96.13%, and the correlation coefficient was also high (Table 2). Therefore, the first four autoregressive parameters *h*_*ik*_(*k*=1,2,…*m*) and the variance *e*_*i*_^2^ of model residuals were chosen as the eigenvectors.

Table 3 shows the average, maximum, and minimum classification rates obtained by the combination of EMD and AR model to extract features (within 4 s after the beginning of visual imagery) and the use of the SVM classifier.

Table 4 shows the average, maximum, and minimum classification rates obtained by using the HHT, the AR, and the combination of the EMD and the AR model to extract features (0–4 s after the beginning of VI tasks) via the SVM classifier.

Figure 3 shows the IMF obtained by EMD of EEG signals during VI tasks. It can be seen from Figure 3 that the EEG signal was decomposed into eight IMF components.

Figure 4 shows curves of classification accuracies as a function of time obtained by the HHT, the AR model, and the combination of the EMD and the AR model. The results of Figure 4(a) show that the classification curve of the test set at 0.0–4.0 s was generally stable and that the classification accuracy was the lowest at the beginning of the test. There was a maximum value between 0.3 and 0.8 s, a maximum value between 0.8 and 2.8 s, a maximum value between 2.8 and 3.5 s, and a maximum value between 3.5 and 4.0 s that tended to be stable.  Figure 4(b) shows that the overall fluctuation of the classification curve of the test set was within 0.0–4.0 s and was relatively large, and the classification accuracy was the lowest at the beginning of the test and tended to decline within 0.0–1.0 s, with a maximum within 1.0–1.5 s, a minimum within 1.5–2.5 s, and a decline within 2.5–4.0 s. The results of Figure 4(c) show that the classification curve of the test set in 0–4 s tended to be stable as a whole, rising at 0.0–1.0 s, remaining stable at 1.0–3.0 s, and rising at 3.0–4.0 s.

## 4. Discussion

Many MI-BCI studies using EEG signals for analysis have been published. Although some elucidations have been made with this approach, MI tasks are not easy to acquire and control, as many subjects are incapable of performing MI tasks. Compared with the large volume of MI-BCI studies, fewer VI-BCI studies have been conducted. Importantly, VI tasks are easier to acquire and control compared to MI tasks.

In this study, visualizations of static and moving pictures were selected as VI task pairs. We hypothesized that the characteristic EEGs induced by these two different VI tasks would be separable. The most significant difference between the EEG signals induced by the two VI tasks appeared in the *α* band of FP2 and F8 (Table 1). The variance contribution rate of the first four IMF components reached 96.13%, and the correlation coefficient was high (Table 2). The features extracted between the two VI-task-based EEG signals by the combination of EMD and AR model could be distinguished to a certain extent (average classification accuracy: 78.40 ± 2.07%; Table 3). Therefore, the two different VI tasks in this study were separable. Our future work will aim to further develop feature-extraction and classification methods to potentially improve this classification accuracy.

For the extraction of VI features in VI-BCIs, previous studies have mainly used EEG power-spectrum estimations or frequency bands [1, 4, 8, 9]. In [33], Llorella et al. created two different models of neural networks such as densely connected neural networks (NN) and convolutional neural networks (CNN) through genetic algorithms (GA) for classification. The result obtained is a 60.5% success rate for the five mental states using the CNN + GA technique. In this study, the HHT, the AR model, and a combination of the EMD and the AR model were used to extract features, while SVM was used to classify the EEG signals induced by VI task pairs. According to the results in Table 4, the average classification accuracy of HHT was 11.85% higher than that of the AR model, which showed that the former was better than the latter. The average classification accuracy of the combination of the EMD and the AR model was 10.26% and 22.11% higher than that of the HHT and AR model, respectively, which showed that this combination was better than the HHT or AR model alone. According to the results in Figure 4, the combination of EMD and the AR model yielded a better classification accuracy curve than did the HHT or AR model alone.

Table 5 shows the VI tasks (paradigm), feature-extraction method, classification method, and classification accuracy in VI-BCI studies. In the present study, the average classification accuracy of VIs of moving and static pictures was 26.4% higher than that of Kosmyna et al. and 22.4% higher than that of Neuper et al. We speculated that the VI tasks designed by Kosmyna et al. being all static led to poor separability of the VI-evoked EEG signals. The VI adopted by Neuper et al. induced certain difficulties in hand movements, which led to poor separability of the VI-evoked EEG signals. However, the methods of feature extraction and classification in these studies were different from one another.

The average classification accuracy of this study was 6.2% lower than that of Koizumi et al. which used three types of VI tasks of an UAV moving in three planes (up/down, left/right, front/back). Our present classification accuracy was also 9.24% lower than that of Sousa et al. that used three types of VI tasks of visual imagery: static points; dynamic points moving vertically up and down in two directions; and dynamic points moving up and down, as well as left and right (four directions). Compared with that of Koizumi and Sousa, the classification accuracy of our study was lower. We speculate that since the VI tasks designed by Koizumi and Sousa were dynamic, the VI-evoked EEG signals were more separable. However, the feature-extraction methods of their study and our study were different from one another.

The present study was an off-line VI-BCI study. There are more improved artificial neural networks used in motor task recognition based EEG signals which provided favorable results [34, 35]. To this end, our future work will include the following: (1) online verification and improvement of the proposed methods; (2) further improvement of the VI-BCI experimental paradigm (e.g., new VI tasks); and (3) for the VI-BCI experimental paradigm, further development of effective feature-extraction and classification methods based artificial neural networks.

## 5. Conclusions

This study was aimed at determining classification accuracies of different VI tasks reflected in EEG signals. In order to improve the separability between VI-evoked EEG characteristics, a new paradigm of VI tasks involving visualization of both moving and static pictures was used. We found that the most significant difference between the VI-evoked EEG signals appeared in the *α* band of FP2 and F8. The results showed that the combination of the EMD and the AR model yielded an average classification accuracy of 78.40% ± 2.07%, which was better than that of HHT or the AR model alone. Therefore, it is expected that the recognition of VI of moving and static pictures based on EEGs can be used as a BCI strategy. Additionally, our findings may provide ideas for the construction of a new online real-time VI-BCI with few channels (e.g., FP2 and F8).

## Figures and Tables

**Figure 1:** Two visual imagery tasks used in this study. (a) The subject was instructed to imagine a static star (static picture). (b) The subject was instructed to imagine a star moving to the right (dynamic picture). The dotted arrow in panel b indicates the direction of movement.

**Figure 2:** The timing of a single trial.

**Figure 3:** Each IMF after EMD of EEGs during visual imagery.

**Figure 4:** Classification accuracy over time. (a) HHT was used to extract the curve of classification accuracy varying with time. (b) The AR model was used to extract the curve of classification accuracy varying with time. (c) A combination of EMD and AR model was used to extract the curve of classification accuracy varying with time.

**Table 1:** *t*-test values and visual imagery variance analysis of *p* values for each frequency band of the eight EEG electrode channels.

*t*-test	Delta	Theta	Alpha	Beta	Gamma	ANOVA	
						d*f*	*p*
FP2	0.057	0.623	0.001^*∗∗∗*^	0.065	0.084	3	0.000^*∗∗∗*^
F8	0.124	0.386	0.001^*∗∗∗*^	0.072	0.245	3	0.001^*∗∗∗*^
C3	0.172	0.045^*∗*^	0.023^*∗*^	0.469	0.190	3	0.020
Cz	0.579	0.452	0.008^*∗∗*^	0.754	0.312	3	0.572
C4	0.422	0.325	0.653	0.164	0.270	3	0.023
O1	0.026^*∗*^	0.830	0.035^*∗*^	0.226	0.459	3	0.572
Oz	0.376	0.962	0.274	0.395	0.731	3	0.970
O2	0.076	0.631	0.938	0.339	0.126	3	0.136

Note. ^*∗*^*p* < 0.05, ^*∗∗*^*p* < 0.01, and ^*∗∗∗*^*p* < 0.001.

**Table 2:** Variance contribution rates and correlation coefficients of all IMF components.

IMF components	1	2	3	4	5	6	7	8
Variance contribution rates (%)	57.1652	17.5349	14.1053	7.3225	1.4372	1.0732	0.7628	0.5989
Correlation coefficients	0.7526	0.4932	0.4021	0.2136	0.0034	0.0023	0.0013	0.0006

**Table 3:** Classification accuracy of feature extraction using EMD and AR model.

Sub	Average	Maximum	Minimum
1	79.40	80.13	63.02
2	76.12	73.33	57
3	77.27	87	62.45
4	81.23	86	60.75
5	79.28	83	56
6	77.43	85	65.34
7	82.55	81.33	59.36
8	69.22	88	62
9	69.50	84.33	63.23
10	31.70	46	26.66
11	81.79	85	48.33
12	78.37	86.33	68.33
13	77.99	83.48	63.24
14	41.20	60	31.66
15	78.23	87	68.33
16	35.90	41.66	30
17	77.52	76.66	63.33
18	80.20	83.29	61.71

**Table 4:** Average, maximum, and minimum classification rates obtained by the HHT, the AR, and the combination of the EMD and the AR model.

Feature-extraction method	HHT	AR	EMD + AR
Classification time period (s)	0–4	0–4	0–4
Average (%)	68.14 ± 3.06	56.29 ± 2.73	78.40 ± 2.07
Maximum (%)	78.33	71.67	87
Minimum (%)	53.33	30	48.33

**Table 5:** VI task (paradigm), feature-extraction method, classification method, and classification accuracy in VI-BCI research.

Author	VI tasks	Feature-extraction method	Classification method	Classification accuracy
Kosmyna et al.	Flower; hammer	Power spectrum	SpecCSP	52%
Neuper et al.	Visualizing the movement of one's hand; resting state	Frequency band	DSLVQ	56%
Koizumi et al.	UAV moves in three planes (up/down, left/right, front/back)	PSD	SVM	84.6%
Sousa et al.	Static point; dynamic point moving vertically in two directions; and dynamic point moving vertically in four directions	Power-spectrum energy	SVM	87.64%
This research	Static star and star moving right	HHT, AR model, and EMD + AR	SVM	HHT: 68.14 ± 3.06% AR: 56.29 ± 2.73% EMD + AR: 78.40 ± 2.07%

## Data Availability

The data used to support the findings of this study are available from the corresponding author upon request.
